# An Efficient Parallelized Ontology Network-Based Semantic Similarity Measure for Big Biomedical Document Clustering

**DOI:** 10.1155/2021/7937573

**Published:** 2021-11-09

**Authors:** Meijing Li, Tianjie Chen, Keun Ho Ryu, Cheng Hao Jin

**Affiliations:** ^1^College of Information Engineering, Shanghai Maritime University, Shanghai 201306, China; ^2^Data Science Laboratory, Faculty of Information Technology, Ton Duc Thang University, Ho Chi Minh 700000, Vietnam; ^3^Biomedical Engineering Institute, Chiang Mai University, Chiang Mai 50200, Thailand; ^4^Department of Computer Science, College of Electrical and Computer Engineering, Chungbuk National University, Cheongju 28644, Republic of Korea; ^5^ENN Research Institute of Digital Technology, Beijing 100096, China

## Abstract

Semantic mining is always a challenge for big biomedical text data. Ontology has been widely proved and used to extract semantic information. However, the process of ontology-based semantic similarity calculation is so complex that it cannot measure the similarity for big text data. To solve this problem, we propose a parallelized semantic similarity measurement method based on Hadoop MapReduce for big text data. At first, we preprocess and extract the semantic features from documents. Then, we calculate the document semantic similarity based on ontology network structure under MapReduce framework. Finally, based on the generated semantic document similarity, document clusters are generated via clustering algorithms. To validate the effectiveness, we use two kinds of open datasets. The experimental results show that the traditional methods can hardly work for more than ten thousand biomedical documents. The proposed method keeps efficient and accurate for big dataset and is of high parallelism and scalability.

## 1. Introduction

Recently, researchers pay much attention to semantic information discovery. Semantic data mining has been introduced into various fields of text mining, such as text clustering [1, 2], text classification [3, 4], information extraction [5–7], named entity recognition [8–10], and sentiment analysis [11–13]. Machine learning is the most commonly used method in text mining. In the latest research for text classification, ensemble strategy is often applied, which can capture multiple characteristics from complex text data [14–17].

For text clustering, with the continuous growth of data scale, it poses a challenge for people to mine information hidden in big text data. Since the similarities between texts are required before clustering, it is imperative to explore effective methods of computing similarity under the big data background [18].

Document clustering is an important application in the text clustering domain which helps people navigate the interested documents conveniently [19, 20]. Detecting the text similarity is of great importance in document clustering, which directly affects the performance of clustering. Numerous studies about similarity detection have been proposed, including vector-based [21–23] and ontology-based [24, 25]. The vector-based methods change the text into vector representation and then view the cosine similarity between vectors as the text similarity. The ontology-based methods use a structural knowledge representation network to describe the meanings and relationships of concepts. Since the vector-based methods ignore the semantic information between words, the ontology-based method attracts much attention at present [26].

An ontology is a hierarchical structure in which concepts are represented as nodes. And the nodes are connected with some relationships such as “is a” and “part of.” Thus, the semantic similarity between concepts can be quantified in an ontology by detecting the node correlation in the structure. Existing ontology-based semantic similarity measurements can be divided into four categories. The first type is path-based, which takes the path distance between nodes in the structure as a measure of correlation. Bulskov et al. [27] used the path length between two nodes in the ontology. The path length is computed by the edges connecting the nodes. Wang [28] gave precomputed weights to edges on the basis of Buskov's method. The second type is information content (IC) based. Information content is the amount of information that a concept expresses, which can be computed from the ontology and corpus. The more a concept occurs, the less information content it has. Resnik [29] took the IC value of the least common ancestor (LCA) of the two nodes as the semantic similarity. Lin [30] extended the method by normalizing the IC value of the LCA using the IC value of both nodes. The third type is depth-based. Leacock and Chodorow [31] and Li et al. [32] took the depth of nodes in the ontology into account since the depth of nodes represents the information specificity. The fourth type is hybrid. Hybrid methods use more than one class of information. Jiang and Conrath [33] and Zhao and Wang [34] combined the IC and depth of nodes to compute the similarity.

In the domain of biomedical text mining, Medical Subject Headings (MeSH) is one of the most commonly used ontologies, which contains 29,638 MeSH headings arranged hierarchically in a tree structure by 2020 [35, 36].

Nowadays, with the rapid development of biomedicine, the amount of biomedical literature grows rapidly. Even if people narrow the search scope, a lot of literatures are retrieved. For instance, over the past five years, PubMed (http://pubmed.ncbi.nlm.nh.gov) has indexed more than 900 hundred biomedical citations by querying “cancer” in all fields. In addition, due to the complexity of ontology-based semantic similarity calculation, computing semantic similarity between a big number of documents leads to low efficiency. Our experiments show that the existing methods can hardly work with more than ten thousand documents. However, clustering is more valuable when the amount of data is larger.

To solve these problems, we proposed a method on the basis of Hadoop MapReduce. Hadoop is a framework that allows for distributed processing across clusters of computers. MapReduce is a module of Hadoop, allowing the parallel processing of large data sets. Traditionally, the document similarity is computed pair by pair, which causes redundant computation. The proposed method parallelizes the process of computing document similarity for the purpose of reducing the computational redundancy and increasing the amount of data that can be processed.

## 2. Materials and Methods

### 2.1. Definition

The set of documents to be clustered is denoted by *D*(*D* = {*d*_1_, *d*_2_, ⋯, *d*_*n*_}). Similarly, the set of MeSH headings is denoted by *M*(*M* = {*m*_1_, *m*_2_, ⋯, *m*_*n*_}). In this article, we define the MeSH headings as the semantic features of biomedical documents since the MeSH headings describe the subject of each article in MEDLINE. Thus, we use a set of MeSH headings to represent a document: *d* = {*m*_*k*_1__, *m*_*k*_2__, ⋯, *m*_*k*_*n*__}, where *j* is the index of MeSH headings.

In the MeSH ontology, each MeSH heading is mapped to one or more nodes associated with tree numbers. The deeper the node is, the more specific the information is. The MeSH Tree nodes are denoted by *V*(*V* = {*v*_1_, *v*_2_, ⋯, *v*_*n*_}). Similarly, a set of nodes are used to represent a MeSH heading: *m* = {*v*_*j*_1__, *v*_*j*_2__, ⋯, *v*_*j*_*n*__}, where *j* is the index of nodes.

Table 1 shows an example of a document with MeSH headings and corresponding tree number of nodes.

Define Sim(·, ·) a function that outputs the similarity between two inputs. For example, Sim(*v*, *v*′) outputs the similarity between two nodes, and Sim(*m*, *d*) outputs the similarity of a MeSH heading to a document. Define *lca*(*v*, *v*′) outputs the LCA (least common ancestor) of two nodes in the MeSH ontology.

In MapReduce programming model, data is represented as key-value pairs. The key-value pair is denoted by <*k*, *v*>. Generally, a MapReduce task mainly consists of three stages: map, shuffle, and reduce. The input file is first divided into multiple splits through the input format, and each split will be assigned a map task. The map task processes the input file line by line and outputs intermediate key-value pairs: <*k*_1_, *v*_1_>. Shuffle is a process after the map task. Shuffle copies data from the map task to the reduce task, sorts the data according to the key value, and aggregates data with the same key: <*k*_2_, list(*v*)>. The reduce task processes the shuffled data line by line and then outputs new key-value pairs: <*k*_3_, *v*_3_>.

### 2.2. Overview

The workflow of the proposed method is as Figure 1 shows. The input is the biomedical documents, and the output is the document cluster. The details are as follows:

1. *Preprocessing*. The first step is to extract the semantic features of each document. The second step is to transform the data to put together documents that have the same semantic feature by using MapReduce
2. *MapReduce-Based Semantic Similarity Calculation*. Calculate the MeSH heading similarity in advance and then calculate the document similarity with the average maximum match
3. *Document Clustering*. Apply the cluster algorithm over the document similarity. In this article, we perform *K*-means, agglomerative clustering, and spectral clustering, respectively, over the document similarity

### 2.3. Preprocessing

In MEDLINE, each document is associated with a unique PubMed ID (PMID) and is tagged with several MeSH headings. Since the MeSH headings describe the subject of the documents, the MeSH headings can be viewed as semantic features. Furthermore, the semantic similarity between documents can be represented by the semantic similarity between the sets of MeSH headings. Zhu et al. [37] and Zhou et al. [38] have proved the feasibility of this method. Therefore, we first extract the corresponding MeSH headings of documents through Efetch in NCBI. To put together documents that have the same semantic features, we transform the input document denoted by “*d*_*k*_#*m*_*k*_1__, *m*_*k*_2__, *m*_*k*_3__” into the format “*m*_1_#*d*_1_, *d*_2_, *d*_4_” which means that the documents ^"^*d*_1_,” “*d*_2_,” and “*d*_4_” contain the same MeSH heading “*m*_1_.” The output is denoted as <*m*, list(PMID)>, where *m* is a MeSH heading.

The data transformation algorithm is as follows:

### 2.4. Semantic Similarity Calculation

To compute the semantic contribution of each MeSH heading to the document, we use Wang's average maximum match (AMM) strategy [39]. In Wang's study, Wang used AMM strategy to compute the semantic similarity between two sets of Gene Ontology (GO) terms. Since the AMM strategy is able to accurately detect the similarity between sets of semantic features, we applied AMM strategy to compute the semantic similarity between two sets of MeSH headings. The AMM strategy is defined as follows:

(1) $$\begin{array}{c} \text{Sim}\left(d,d^{\prime }\right)=\frac{\sum_{m\in d}\text{S}\text{im}\left(m,d^{\prime }\right)+\sum_{m\prime \in d\prime }\text{S}\text{im}\left(m^{\prime },d\right)}{\text{MeSHNumber}\left(d\right)+\text{MeSHNumber}\left(d^{\prime }\right)}, \end{array}$$

(2) $$\begin{array}{c} \text{Sim}\left(m,d\right)=\max_{m^{\prime }\in d}\text{Sim}\left(m,m^{\prime }\right), \end{array}$$

(3) $$\begin{array}{c} \text{Sim}\left(m,m^{\prime }\right)=\frac{\sum_{v\in m}\text{S}\text{im}\left(v,m^{\prime }\right)+\sum_{v\prime \in m\prime }\text{S}\text{im}\left(v^{\prime },m\right)}{\text{NodeNumber}\left(m\right)+\text{NodeNumber}\left(m^{\prime }\right)}, \end{array}$$

(4) $$\begin{array}{c} \text{Sim}\left(v,m\right)=\max_{v^{\prime }\in m}\text{Si}{\text{m}}^{\text{sem}}\left(v,v^{\prime }\right), \end{array}$$

where NodeNumber() returns the node number of the MeSH heading, and MeSHNumber() returns the MeSH heading number of the document. The semantic measure is optional. The measures used in this paper are as follows:

(1) SP [27]
  (5) $$\begin{array}{c} \text{Si}{\text{m}}^{\text{SP}}\left(m,m^{\prime }\right)=\frac{L_{\max}\left(m,m^{\prime }\right)-L_{\min}\left(m,m^{\prime }\right)}{L_{\max}\left(m,m^{\prime }\right)}, \end{array}$$
  where *L*_max_(*m*, *m*′) returns the longest path length, and *L*_min_(*m*, *m*′) returns the shortest path length.
(2) WP [28]
  (6) $$\begin{array}{c} \text{Si}{\text{m}}^{\text{WP}}\left(v,v^{\prime }\right)=\frac{2*\text{depth}\left(lca\left(v,v^{\prime }\right)\right)}{\text{depth}\left(v\right)+\text{depth}\left(v^{\prime }\right)}, \end{array}$$
  where depth(*v*) returns the tree depth of the node.
(3) LC [31]
  (7) $$\begin{array}{c} \text{Si}{\text{m}}^{\text{LC}}\left(m,m^{\prime }\right)=1-\frac{\log\left(1+L_{\min}\left(m,m^{\prime }\right)\right)}{\log\left(1+2D\right)}, \end{array}$$
  where *D* is the maximum depth of the heading in MeSH ontology.
(4) Res [29]
  (8) $$\begin{array}{c} \text{Si}{\text{m}}^{\text{Res}}\left(v,v^{\prime }\right)=\text{IC}\left(lca\left(v,v^{\prime }\right)\right). \end{array}$$
(5) Lin [30]
  (9) $$\begin{array}{c} \text{Si}{\text{m}}^{\text{Lin}}\left(v,v^{\prime }\right)=\frac{2*\text{IC}\left(lca\left(v,v^{\prime }\right)\right)}{\text{IC}\left(v\right)+\text{IC}\left(v^{\prime }\right)}. \end{array}$$
(6) Sch [40]
  (10) $$\begin{array}{c} \text{Si}{\text{m}}^{\text{Sch}}\left(v,v^{\prime }\right)=\frac{2*\text{IC}\left(lca\left(v,v^{\prime }\right)\right)}{\text{IC}\left(v\right)+\text{IC}\left(v^{\prime }\right)}*\left(1-\exp\left(-\text{IC}\left(lca\left(v,v^{\prime }\right)\right)\right)\right), \end{array}$$
  (11) $$\begin{array}{c} \text{IC}\left(v\right)=H\left(v\right)*\left(1-\frac{\log\left(\left|C\left(v\right)\right|+1\right)}{\log\left(T_{\text{total}}\right)}\right). \end{array}$$

IC(*v*) returns the IC value of the node. *H*(*v*) returns the depth of the node in the ontology. *C*(*v*) is the set of the children of the node, and *T*_total_ is the total node number of the ontology.

We use SORA [41] to calculate the IC value. It is an ontology structure-based method, outperforming the corpus-based method on computation time.

According to AMM, semantic similarity calculation is divided into MeSH heading similarity calculation and document similarity calculation. Since the MeSH heading similarity is frequently used when computing the document similarity, we calculate the similarity of all pairs of extracted MeSH headings in advance. The MapReduce-based MeSH heading similarity calculation algorithm is as follows:

Traditionally, document similarity is calculated pair by pair, leading to large computational cost, which is the main reason why the existing methods can hardly work with a large number of documents. To make the AMM applied to the parallelization condition, we designed a MapReduce-based algorithm to calculate the document similarity in parallel. In this method, the similarity contribution of a MeSH heading to a document is viewed as a basic computation element. By splitting the semantic similarity between documents into the aggregation of multiple heading-to-document similarity denoted as sim(*m*, *d*), we realized the parallel computation of the document similarity. In addition, for each line of input, we directly output the semantic similarity of the MeSH heading to other documents, avoiding redundant computation. The algorithm is as follows, and an example is given in Figure 2:

Supposing that the number of documents is *n*, average MeSH headings number of documents is *m*, the total number of MeSH headings is *k*, and the time complexity of the traditional method is *O*(*m*^2^*n*^2^). For the proposed MapReduce-based algorithm, the time complexity of map stage is *O*(*kmn*), and the time complexity of reduce stage is *O*(*n*^2^).

### 2.5. Document Clustering

Spectral clustering [42, 43], agglomerative clustering [44, 45], and *K*-means [46, 47] are commonly used in text clustering. Spectral clustering is based on graph, which transforms the clustering problem into the optimal partition problem of a graph by treating each document as the vertex of the graph and the similarity between documents as the edge weight. The clusters are obtained by cutting the graph according to some rules such as Ncut [48] and Mcut [49]. Agglomerative clustering treats each document as a cluster first and then merges the most similar cluster repeatedly. *K*-means is carried out through multiple iterations. In each iteration, each document is divided into the most similar cluster until the cluster no longer changes. In this paper, these three clustering algorithms are performed, respectively, over the document similarity.

### 2.6. Data

For the analysis of multiangle, two kinds of datasets were applied in this experiment. One is a small and labelled dataset named SL used for verifying the accuracy of the proposed method. The other one is large and unlabelled dataset named LUs, being used for testing the efficiency of the method when dealing with a large number of documents.

SL is generated from Text REtrieval Conference (TREC) genomics track 2005, which contains biomedical documents with 50 topics. In TREC genomics track, each document is judged as definitely relevant (DR), possibly relevant (PR), or not relevant (NR) to the topic. We remove the PR and NR documents, reserving DR documents.

When generating the data set, we referred to the practice of Gu et al. [50]. To avoid small clusters, we remove the topics that have less than 10 documents. Furthermore, we remove the documents that are relevant to 2 or more topics. Finally, the dataset of 2,317 documents with 24 topics were obtained. We randomly selected documents of 3-12 topics to generate 100 different datasets.  Table 2 shows the summary of these datasets.

LUs include six datasets randomly extracted 10000 to 60000 documents from PubMed, covering more than 20000 different MeSH headings. For each dataset, we mark it with the number of documents, such as LUs-10000 and LUs-20000.  Table 3 is the summary of the dataset LUs.

### 2.7. Evaluation Criteria

In the experiment, the performance is evaluated by comparing the predicted label and the true label. We take Normalized Mutual Information (NMI) as the evaluation index, since it has been proved that NMI outperforms many other clustering evaluation indexes [40]. The NMI formula [41] is defined as follows:

(12) $$\begin{array}{c} \text{NMI}=\frac{\sum_{h,l}n_{h,l}\log\left(n\cdot n_{h,l}/n_{h}n_{l}\right)}{\sqrt{\left(\sum_{h}n_{h}\log\left(n_{h}/n\right)\right)\left(\sum_{l}n_{l}\log\left(n_{l}/n\right)\right)}}, \end{array}$$

where *n* is the total number of documents to be clustered, *n*_*h*_ is the number of documents with true class *h*, *n*_*l*_ is the number of documents with predicted class *l*, and *n*_*h*,*l*_ is the number of documents with true class *h* and predicted class *l*.

NMI ranges from 0 to 1. A high NMI value means the strong correlation between the predicted label and the true label.

### 2.8. Experimental Environment

The hardware and software details of each computer are shown in the following table.

The experimental environment is a Hadoop cluster composed of five computers with the same configuration.

## 3. Results and Discussion

### 3.1. Optimization of MapReduce Job Settings

Before testing the efficiency of the proposed method with a large number of documents, MapReduce job settings are optimized according to the characteristics of the proposed method since the job settings have a great impact on task execution [51]. It can be easily found that the input and output of the proposed method are very compact, while a lot of intermediate key-value pairs are generated in the Map task during MapReduce-based semantic similarity calculation, which will generate much data to be sorted and aggregated in Shuffle. Therefore, according to the MapReduce optimization principle of multiset homomorphisms proposed by Dorre et al. [51], we increase the number of reduce tasks to enhance the parallelism and add the combiner used to aggregate the data before shuffle.

As is shown in Figure 3, on the dataset LUs-10000 with Resnik measure, the elapsed time of map is reduced from 0.5 minutes to 0.45 minutes, the elapsed time of shuffle is reduced from 2.77 minutes to 1.3 minutes, and the elapsed time of reduce is reduced from 2.05 minutes to 0.56 minutes. The result shows that the optimization reduces the intermediate data to be shuffled and promotes the efficiency of reduce, effectively decreasing the computation time. And we used the same optimized job settings in the following experiments.

### 3.2. Evaluation of Clustering and Computation Efficiency

In the experiment, the proposed method was conducted with six semantic measures and three cluster algorithms. Then, we compared the traditional method with the proposed method on both computation time and NMI. Tables 5 and 6 show the results.

- Computational efficiency

For the small dataset SL, the traditional method takes more than an hour, while the proposed method takes no more than 3 minutes with the cluster of five computers. For the big dataset LUs-10000, the traditional method can hardly work due to the big data, while the proposed method keeps efficient. Various semantic measures are available in this method, and the IC-based methods take less time than other methods.

(B) Clustering validation

For the spectral clustering, the highest NMI of 0.647 is achieved with Resnik. For the *K*-means, the highest NMI of 0.526 is achieved with Lin. For the agglomerative clustering, the highest NMI of 0.591 is achieved with Resnik. The result reveals that the information content-based measure (Resnik and Lin) outperforms other semantic measures, and spectral cluster performs better than the other two cluster algorithms. The highest NMI is obtained by Resnik measure and spectral clustering algorithm. Compared with the result in Zhu et al.'s study [37] where the same data and evaluation criteria were used, NMI of the proposed method is slightly increased, implying that the proposed method greatly improves the computational efficiency without decreasing the clustering accuracy.

### 3.3. Speedup and Elapsed Time with Different Cluster Node Number

To study the parallelism of the method, the proposed method was performed with different cluster node number on dataset LUs of 10000 documents.  Figure 4 shows that the elapsed time goes down from 12.63 minutes to 2.31 minutes, and the speedup goes up almost linearly from 1 to 5.45 as the cluster nodes increase, implying that the proposed method is of high parallelism, and increasing nodes will improve the computation time effectively.

### 3.4. Computation Time with More Documents

In this section, the experiment was performed on the dataset LUs to observe the trend of the elapsed time and the proportion of each stage in the MapReduce job.  Figure 5 shows that the proposed method remains effective when processing a big number of documents. As the documents increase, the elapsed time of map and reduce grows slowly while the elapsed time consumed in shuffle grows rapidly. And shuffle accounts for the largest proportion of computation time in all MapReduce tasks. The result reveals that the sort and copy of data become the key factor to the computation time when processing a big number of documents.

## 4. Conclusions

In this paper, we developed an efficient ontology-based semantic similarity measure for big document data clustering. Traditionally, the semantic similarity between documents is computed in pairwise, which can hardly work with a big number of documents. To solve the problem, we developed a MapReduce-based method to process the data in parallel. By splitting the document similarity into the aggregation of multiple heading-to-document similarity, the proposed method avoids the redundant computation and is available to process a big number of documents in a short time. Additionally, according to the experiment results, it can be concluded that the proposed method is of high parallelism and scalability, implying that more documents can be processed as long as we increase the cluster nodes, upgrade the hardware of computers, and optimize the job settings properly. In this work, both semantic measure and the cluster algorithm are optional, which depend on the datasets and the ontology. For the TREC 2005 genomics track dataset and MeSH ontology, the spectral algorithm and the semantic measure of Resnik perform better than other parameters. Furthermore, the proposed method is not limited to biomedical documents and MeSH ontology. The proposed method can also work in the situation of combining semantic similarity from different semantic features.

## Figures and Tables

**Figure 1:** The workflow of the proposed method.

**Figure 2:** An example of MapReduce-based data transformation and semantic similarity calculation.

**Figure 3:** The result of MapReduce job optimization.

**Figure 4:** The trend of speedup and computation time with increasing cluster nodes.

**Figure 5:** Computation time of map, shuffle, and reduce on dataset LUs.

**Algorithm 1:** Algorithm of MapReduce-based data transformation.

**Algorithm 2:** Algorithm of MapReduce-based MeSH heading similarity calculation.

**Algorithm 3:** Algorithm of MapReduce-based document similarity calculation.

**Table 1:** An example of a biomedical document (PMID: 10496010) with corresponding MeSH headings and tree number of nodes.

MeSH heading	Tree number
DNA repair	G02.111.222
	G05.219
Genetic diseases, inborn	C16.320
Humans	B01.050.150.900
	.649.313.988.400
	.112.400.400

**Table 2:** Summary of the dataset SL.

	Documents	Classes	Unique MeSH headings	Total MeSH headings
Min	51	3	387	1619
Max	1619	12	2502	25631
Mean	689	7.5	1458	2502

**Table 3:** Summary of the dataset LUs.

	Documents	Unique MeSH headings	Total MeSH headings
Min	10000	14499	123347
Max	60000	25742	731089
Mean	35000	21540	427731

**Table 4:** Configuration of computers.

Configuration	Details
OS	Centos 7
CPU	I5-6500, 3.2 GHz
HDD	1 TB, 7200 rpm
RAM	8 G
Hadoop	Hadoop 3.1.3
JDK	1.8.0_252

**Table 5:** Computation time (minutes) of the traditional and proposed method with different semantic measures (“/” means cannot work).

Method	Dataset: SL						Dataset: LUs-10000					
	SP	WP	LC	Res	Lin	Sch	SP	WP	LC	Res	Lin	Sch
Traditional	68.9	66.35	67.9	61.15	64.8	66.25	/	/	/	/	/	/
Proposed	2.87	1.02	1.42	1.15	0.95	1.17	10.21	3.43	5.02	2.31	3.30	3.77

**Table 6:** NMI (Average ± Standard Deviation) on dataset SL with different cluster algorithms and semantic measures.

Cluster algorithm	SP	WP	LC	Resnik	Lin	Sch
Spectral clustering	0.579 ± 0.126	0.549 ± 0.132	0.574 ± 0.130	0.647 ± 0.124	0.617 ± 0.111	0.527 ± 0.124
*K*-means	0.490 ± 0.140	0.495 ± 0.131	0.491 ± 0.134	0.511 ± 0.176	0.526 ± 0.158	0.520 ± 0.123
Agglomerative clustering	0.524 ± 0.123	0.551 ± 0.145	0.533 ± 0.124	0.591 ± 0.116	0.582 ± 0.135	0.523 ± 0.126
Zhu	/	0.568 ± 165	0.565 ± 0.169	/	0.620 ± 0.161	/

## Data Availability

The data are available from Text REtrieval Conference (TREC, https://trec.nist.gov/) and PubMed (https://pubmed.ncbi.nlm.nih.gov/).
